RETRACTED

# Oral Administration of Brain Protein Combined With Probiotics Induces Immune Tolerance Through the Tryptophan Pathway

**DOI:** 10.3389/fnmol.2021.634631

**Published:** 2021-05-28

**Authors:** Yongxin Hou, Lixia Xu, Sirong Song, Weijia Fan, Qiaoli Wu, Xiaoguang Tong, Hua Yan

**Affiliations:** ^1^School of Medical, Nankai University, Tianjin, China; ^2^Tianjin Neurosurgical Institute, Tianjin Key Laboratory of Cerebrovascular and Neurodegenerative Diseases, Tianjin Huanhu Hospital, Tianjin, China; ^3^Graduate School of Tianjin Medical University, Tianjin, China; ^4^Department of Neurosurgery, Tianjin Huanhu Hospital, Tianjin, China

**Keywords:** TBI, immune tolerance, probiotics, tryptophan, IDO, 5-HT

## Abstract

Excessive inflammation leads to secondary immune damage after traumatic brain injury (TBI). The intestinal mucosa is a key component of immune tolerance due to gut-brain axis regulation, but the curative effect is not optimal. Intestinal dysfunction impairs the establishment of immune tolerance in patients with TBI. Therefore, we orally administered brain protein (BP) combined with probiotics to induce immune tolerance and explored the mechanism by which the homeostasis of the microbiota contributes to the enhancement of curative effects by BPs. Herein, we demonstrated that patients with TBI and surgical brain injury (SBI) models of rats had obvious dysbiosis. Notably, the intestinal barrier, proinflammatory cytokines, and activation of microglia demonstrated that excessive inflammatory damage was better controlled in the combined group (oral administration of BP combined with probiotics) than in the BP group (oral administration of BP). Fundamentally, tandem mass tag (TMT)-based quantitative proteomics analysis revealed that BP and probiotics preferentially affect Try-related pathways. A series of experiments further confirmed that Indoleamine 2,3 dioxygenase (IDO)/Kynurenine (Kyn)/Aryl hydrocarbon receptor (AhR) expression was high in the BP group, while Tryptophan hydroxylase 1(TpH1)/5-hydroxytryptamine (5-HT) only changed in the combined group. This study suggests that probiotics can enhance the efficacy of oral BP-induced immune tolerance through the Try pathway.

## Introduction

Head injuries and their sequelae have become increasingly important public health issues (Sundman et al., 2017). Immunosuppression therapy and immune tolerance therapy after traumatic brain injury (TBI) have attracted the attention of the academic community. The common physiological and anatomical bases of these conditions involve the destruction of the blood-brain barrier and the exposure of brain tissue, which in turn cause brain tissue antigens to be recognized by the body’s immune system, thereby triggering aggressive autoimmune behavior and resulting in secondary immune damage. Immunosuppressive drugs are used to treat secondary nervous system damage but have important shortcomings, such as high cost, a narrow safety spectrum, and exacerbated infection.

RETRACTED

Through specific immune-tolerant organs or tissues from the body, brain antigen-induced immune tolerance can create a minimal immune response to brain antigens that does not excessively affect the body’s immunity (Tian et al., 2019). Immune tolerance is established in multiple ways, such as the oral administration or injection of autologous brain antigens *via* the thymus and liver, and each method has advantages and disadvantages. However, in terms of the convenience of clinical promotion, the oral administration of autologous brain antigens (derived from necrotic brain tissue and drained cerebrospinal fluid from the brain contusion and laceration) is pivotal, and the intestinal mucosa is a key component of immune tolerance. Although therapy has been proven to be effective in patients with TBI and has been recognized by academia, the efficacy has not reached expectations. After a severe head injury in rats, the intestinal flora is in a severely unbalanced state (Yu et al., 2011); we often observe extremely high incidence rates of diarrhea and stress ulcers in patients with severe TBI in clinical work. Increased intestinal inflammation exerts a key influence on the pathophysiologic processes following injury (Earley et al., 2015). Intestinal wall damage leads to inflammation of the mucosal barrier (Winter et al., 2013; Albenberg et al., 2014; Dickson, 2016); intestinal permeability increases, and substances can aberrantly penetrate the barrier to disrupt normal physiological functions. Such deficits in intestinal permeability typically lead to an innate immune response that underpins chronically elevated levels of inflammation, which are known to promote disease (Turner, 2009; Gallo and Hooper, 2012). Probiotics can fortify the intestinal barrier to mitigate neurotrauma-induced endotoxemia and inhibit systemic dysregulation of the immune system that may otherwise peripherally hyperactivate the brain’s microglia (Lamprecht et al., 2012; de Punder and Pruimboom, 2015).

The mechanisms of immune tolerance by brain proteins (BPs) and the enhancement of immune tolerance by probiotics have not been clarified thus far. In this study, we performed tandem mass tag (TMT)-based quantitative proteomics analysis and revealed that BPs and probiotics preferentially affect Try-related pathways.

## Materials and Methods

### Ethics for Patients and Rats

The patients or their direct relatives were informed of the clinical experimental process and provided written consent. Male adult Sprague–Dawley rats were obtained from the Experimental Animal Center of the Academy of Military Medical Sciences, China. Animals were kept on a 12-h light and dark cycle and housed in sterile vent/rack cages with ad libitum access to food and water at the Animals Center of Huanhu Hospital Tianjin. All methods were performed in accordance with the relevant guidelines and regulations and approved by the Tianjin Key Laboratory of Cerebral Vascular and Neurodegenerative Diseases, China. Laws and rules were strictly obeyed to protect the animals from abuse.

RETRACTED

### Study Population

To conduct a case-control study, we examined two distinct populations matched for age, fat mass and, sex. According to the case-control study, 24 patients with moderate and severe TBI who were admitted to the Brain Trauma Center 2 ward from October 2018 to February 2019 were included in the case group; moreover, 10 healthy volunteers matched for age and sex were selected as the control group. The experimental criteria were as follows: (1) patients with TBI were assessed by a specialist to ensure they met the clinical classification of acute closed-head injury, with a Glasgow scale of less than 12; (2) patients were aged 18–70 and were from northern China and the Han ethnic group; (3) the age and sex of the healthy subjects matched those of the patients; (4) patients were admitted within 48 h after craniocerebral trauma; (5) patients had no history of antibiotic use in the past 1 month; (6) patients had no probiotic and probiotic use in the past 1 month; and (7) all group members signed informed consent forms and allowed collection of stool samples. The exclusion criteria were as follows: (1) cancer, liver and kidney disease, or gastrointestinal bleeding disease affecting intestinal flora; (2) previous gastrointestinal surgery; (3) fecal sample retention; (4) probiotics taken during treatment; (5) other interventions; and (6) other conditions such as autoimmune disease, hypothyroidism, Parkinson’s disease, previous history of stroke, and major trauma in the first 2 months.

### SBI Model Design

Male Sprague–Dawley rats (grade SPF; 220–250 g; Experimental Animal Center of Academy of Military Medical Sciences, China) were randomly selected. A standardized SBI model was used according to previous reports (Wang et al., 2015). Briefly, before surgery, general anesthesia was induced *via* intraperitoneal injection of 0.3 ml/100 g chloral hydrate. The head and manubrium sterni of the rats were shaved. Next, each rat was fixed in a stereotaxic frame, and the sterile skin on the skull was incised along the biparietal suture through a single sagittal incision. A small square of the skull (4 mm diameter) was thinned and removed with a bone drill on the right skull bone 2 mm along the sagittal suture and 1 mm along the coronal suture. A durotomy was performed, and 2 × 3 mm brain tissue was excised by sharp dissection. Hemostasis was confirmed, and the skin was then closed after SBI. BP or BP combined with probiotics was orally administered to the BP and combined groups, respectively.

RETRACTED

### Repeated Freeze-Thaw Method to Extract Brain Protein and Administration of Brain Protein and Probiotics

After intraperitoneal injection of 0.3 ml/100 g of 10% chloral hydrochloride anesthesia, the skin was exposed. The rats were rapidly fixed on a stereotactic apparatus, and the neck was broken. Under aseptic conditions, the scalp was cut sagittally, the skull was separated, and brain tissue was exposed and removed. Then, the small blood vessels and meningeal tissue on the surface were carefully removed, and brain tissue was cut under aseptic conditions, quickly placed at −80°C for 30 min and in a 37°C water bath for 5 min for rewarming, and ground in a rod-shaped grinding mill for full grinding at 4°C. This step was repeated three to five times, and inverted phase-contrast microscopy was used to confirm that there was no brain cellular morphology. The protein concentration was tested by using ultraviolet spectrophotometry; the solution was adjusted to a 5.0 mg/ml concentration with ultrapure water and placed at −20°C (Fan et al., 2014). The rats in the BP and combination groups underwent gavage administration of BP in 4 ml every day. The rats in the combined group underwent gavage administration of live combined Bifidobacterium and Lactobacillus tablets at 500 mg every day.

### Bioinformatics Processing

Using the IonS5TMXL sequencing platform, we merged, applied quality control, and, clustered the 16S rRNA gene reads into operational taxonomic units (OTUs). Taxonomic groups were based on the Green genes DatabaseV.13_8 using a closed reference to perform referenced-based OTU clustering (Edgar, 2010; McDonald et al., 2012). Values for alpha diversity [Chao1 index, Shannon’s index, phylogenetic diversity (PD), whole tree index and observed OTUs], beta diversity (unweighted UniFrac distance metrics) and principal coordinate analysis (PCoA) employed based on the UniFrac metrics were generated by QIIME V.1.9.1. Permutational multivariate analysis of variance was performed to determine if the compositions of microbiota differed between groups. Linear discriminant analysis effect size (LEfSe) was performed to determine the features most likely to explain the differences between groups (Segata et al., 2011).

RETRACTED

### Quantitative Proteomic Analysis of the Colons and Brains of Rats by (TMT) Technology

Brain and colon tissues were prepared, and peptide TMT labeling was performed. All of our data were collected using an Orbitrap Elite mass spectrometer (Thermo Fisher Scientific, San Jose, CA, USA) coupled with a Famos autosampler (LC Packings) and an Accela 600 quaternary liquid chromatography (LC) pump (Thermo Fisher Scientific). Mass spectra were processed using a software pipeline that was developed in-house and is based around the Sequest algorithm. The 1a, 13 MS spectra were converted to XML files using a modified version of ReAdW.exe and then searched against a database including all entries from the human or mouse International Protein Index databases (version 3.6).

### Immunohistochemistry

Rats were anesthetized and sacrificed by perfusion through the heart with 4% paraformaldehyde in PBS (pH 7.4). Brains, small intestine, and colon were removed, postfixed overnight and sectioned by the Department of Pathology, Huanhu Hospital Tianjin. The sections were pretreated with xylene and then incubated with primary antibodies against rat claudin, occludin, and AhR (Abcam) at 4°C overnight. Next, the sections were incubated with complement, HRP conjugate, and DAB (Abcam). Then, the sections were counterstained with hematoxylin. Images were captured by microscopy (Olympus).

### Immunofluorescence

Sections were prepared as described above. The sections were pretreated with xylene, incubated in a liquid sodium citrate repair water bath for heating repair, and then incubated with Iba and GFAP antibodies (Abcam) at 4°C overnight. Then, they were incubated with the secondary antibody staining solution and counterstained with DAPI (Zhongshan). Finally, they were covered with an antifade mounting medium. Images were captured by fluorescence microscopy (Olympus).

### Protein Expression

Protein was extracted from tissues with commercial lysis buffer. Western blotting was performed as described previously (Chen et al., 2017). Primary antibodies against IDO (Abcam) and glyceraldehyde 3-phosphate dehydrogenase (GAPDH, Invitrogen) were used.

### Intestinal Permeability *In vivo*

This measure is based on intestinal permeability to 4,000-Da fluorescent dextran (Sigma-Aldrich, St. Louis, MO, USA) as described previously (Wang et al., 2001). Briefly, 6-h-fasted mice were injected with fluorescein isothiocyanate (FITC)-dextran by gavage (600 mg/kg body wt, 125 mg/ml). After 1 h, 120 μl of blood was collected from the tip of the tail vein. The blood was centrifuged at 4°C and 12,000 *g* for 3 min. Plasma was diluted in an equal volume of PBS (pH 7.4) and analyzed for FITC-dextran concentration with a fluorescence spectrophotometer (HTS-7000 Plus-plate-reader; Perkin Elmer, Wellesley, MA, USA) at an excitation wavelength of 485 nm and an emission wavelength of 535 nm. Standard curves for calculating the FITC dextran concentration in the samples were obtained by diluting FITC-dextran in nontreated plasma diluted with PBS (1:2 [vol/vol]).

RETRACTED

### HPLC-HRMS

For metabolomic analysis, HPLC-HRMS (high-performance liquid chromatography-high-resolution mass spectrometry) was performed with both a 1290 Infinity HPLC coupled to a 6540 Q-ToF mass spectrometer equipped with a Jet Stream ESI interface (Agilent Technologies) and an Ultimate 3000 HPLC coupled to an LTQ-Orbitrap mass spectrometer through an ESI interface (Thermo Scientific). The experiment was accomplished by Shanghai Bioprofile Technology Company, Ltd. for technological assistance in targeted metabolomics experiments.

### Serum Cytokine Concentrations

After induction of general anesthesia, rats were fixed in the supine position, and blood sampling by cardiac puncture was used to sample 1 ml of blood that was injected into the promoting coagulation tube. Following 30 min of incubation at room temperature, the blood sample was centrifuged at 3,500 rpm/min for 15 min. The serum was transferred to an EP tube and stored at 80°C. According to the ELISA kit protocol (Bio-Swamp) plus the TMB color drops, 5-HT, interleukin 6 (IL-6), interleukin 17 (IL-17), and tumor necrosis factor-alpha (TNFα) concentrations were measured at 1, 7, 14, and 21 days postoperatively using an enzyme reader at 450 nm.

### Statistical Analysis

Data are presented as the mean ± SD. Statistical analyses were performed with SPSS software (version IBM SPSS Statistics 22.0), and cartograms were drawn with GraphPad Prism software (version 5.01). One-way ANOVA and LSD tests were used to determine the significance of differences among subgroups. Independent samples *t*-tests were used to compare the differences among the sham, SBI, PC and combined groups. Two-way ANOVA with the Bonferroni *post hoc* test was performed for multiple comparisons. *P* < 0.05 was considered significant.

## Results

### Dysbiosis of Gut Microbiota in Patients With TBI

A total of 10 healthy control volunteers (HCs) and 24 patients with severe or moderate TBI were included in the present study. According to PCoA, the gut microbiome of the TBI group differed significantly from that of the HCs group using the unweighted UniFrac distance (Figure 1A). Alpha diversity indices, including Chao1 and observed OTUs, were markedly increased in the TBI group (*P* < 0.05; Figures 1B,C).

RETRACTED

**Figure 1:** Dysbiosis of gut microbiota patterns in patients with traumatic brain injury (TBI) and healthy controls (HCs). **(A)** Principal coordinate analysis based on unweighted UniFrac distances revealed that the HC bacterial communities clustered separately from the TBI bacterial communities. Each circle represents a single sample, colored by group. The eigenvalues of the principal coordinates PC1 and PC2 were 29.43% and 10.95%, respectively. Differences in beta diversity between HCs and TBI patients were tested by permutational multivariate analysis of variance (Adonis). **(B,C)** Comparison of alpha-diversity indices (Chao1 index and observed operational taxonomic units) between the TBI and HC groups. **Indicates *p* < 0.01 by the Wilcoxon rank-sum test. **(D)** Linear discriminant analysis effect size identified the most differentially abundant taxa between the two groups. TBI-enriched taxa are indicated with a positive LDA score, and taxa enriched in the HC group have a negative score. Only taxa meeting an LDA significance threshold of >4 are shown. **(E)** Relative abundances of *Enterococcus*, *Parabacteroides, Akkermansia, Lachnoclostridium, Bifidobacterium*, and *Faecalibacterium* between the TBI and HC groups. **p < 0.01; and ***p < 0.001 by the Wilcoxon rank-sum test.

To further identify which bacterial taxa differed between the TBI and HC groups, we performed LEfSe analysis and identified six genera showing significant differences (Figure 1D). Moreover, a comparison of the abundance of the predominant genera showed that *Enterococcus*, *Parabacteroides*, *Akkermansia*, and *Lachnoclostridium* were significantly enriched, whereas *Bifidobacterium* and *Faecalibacterium* were depleted in the patients with TBI (Figure 1E).

### Dysbiosis of Gut Microbiota, Alteration of Mucosal Permeability and Activation of Microglia and Astrocytes in SBI Models

To further confirm that TBI caused intestinal dysfunction, we established an surgical brain injury (SBI) model in rats (Figure 2A). Secondary inflammation was accompanied by the activation of IBA-1 and GFAP. Immunofluorescence staining of IBA-1 and GFAP (Figure 2B) indicated that the damage reached the highest level at 7 days after SBI. To further test whether alterations in the gut microbiota can cause the progression of SBI *in vivo*, we collected fecal samples from the SBI models at 3 and 7 days. In this study, with respect to PCoA, the gut microbiome of the SBI group at 3 and 7 days differed significantly from that of the sham group using the unweighted UniFrac distance (Figure 2C). The Chao1 index in the Sham group was significantly higher than that in the SBI group at 3 days (*P* < 0 05; Figure 2D). To identify which bacterial taxa were distinct between the sham and SBI groups at 3 and 7 days, we performed LEfSe analysis and identified three genera showing significant differences (Figure 2E). Moreover, the comparison of the abundance of the predominant genera showed that *Akkermansia* was significantly enriched, whereas *Lactobacillus* and *Parabacteroides* were depleted in the SBI models. We showed a similarity of intestine dysbiosis induced by TBI and SBI (Supplementary Figure 1). Therefore, these results are in accord with earlier clinical experimental results, and we can conclude that brain injury, regardless of TBI or SBI, gives rise to gut dysbiosis. Regarding the mucosal barrier, the results suggest that the barrier-forming tight junction proteins claudin and occludin were expressed at lower levels in the SBI groups than in the sham group; furthermore, the protein expression levels were lower in the SBI group at 3 days than in the other SBI groups (*P* < 0.05; Figure 2F).

RETRACTED

**Figure 2:** Establishment of surgical brain injury (SBI) models and demonstration of dysbiosis and damage to tight junction proteins in the model. **(A)** The process of manipulation of the SBI model. **(B)** Iba and GFAP expression scoring of microglia and astrocytes measured at 3 and 7 days after SBI compared with those of the sham group.** (C)** Principal coordinate analysis based on unweighted UniFrac distances revealing the difference in bacterial communities clustered between the sham and SBI groups at 3 and 7 days. Each circle represents a single sample, colored by group. The eigenvalues of the principal coordinates PC1 and PC2 were 24.85% and 13.51%, respectively. Differences in the beta diversity between the sham and SBI groups at 3 and 7 days were tested by permutational multivariate analysis of variance (Adonis).** (D)** Comparison of alpha-diversity indices (Chao1 index taxonomic units) between the sham and SBI groups at 3 and 7 days. **Indicates *p* < 0.01 by the Wilcoxon rank-sum test. **(E)** Linear discriminant analysis effect size identified the most differentially abundant taxa among the three groups. Only taxa meeting an LDA significance threshold of >3 are shown. Relative abundances of *Lactobacillus, Parabacteroides*, and *Akkermansia* among the three groups. *p < 0.05, **p < 0.01 by the Wilcoxon rank-sum test. **(F)** Representative images of occludin and claudin immunofluorescence staining in the colon and small intestinal tissues.

### Oral Administration of Brain Proteins and Probiotics Benefits Gut Microbiota, Improves Intestinal Barrier Function and Promotes Brain Tissue Repair

Both gut dysbiosis and dysfunction were proven in patients with TBI and the rat model of SBI. Next, we wanted to further confirm whether the oral administration of probiotics could enhance the immune tolerance induced by the oral administration of brain antigen and thus strengthen the efficacy. After we established the SBI models, the BP and combined groups were orally administered brain antigen and brain antigen combined with probiotics every day. The rats in the four groups were sacrificed at 3, 7, and 14 days (Figure 3A).

RETRACTED

**Figure 3:** The results of immune tolerance induced by the oral administration of brain protein (BP) and BP combined with probiotics in the BP and combined groups compared with the Sham, SBI group. **(A)** The rats of the sham, SBI, BP, and combined groups were sacrificed at 3, 7, and 14 days.** (B)** ELISA results of IL-6, TNF-α, and IL-17 among the SBI, BP, and combined groups at 1, 3, 7, and 14 days. **(C)** Iba and GFAP expression scoring of microglia and astrocytes measured at 3 days after SBI compared with those of the BP and combined groups. **(D)** Comparison of alpha-diversity indices (Chao1 index taxonomic units) among the sham, SBI, BP, and combined groups at 3 days. **Indicates *p* < 0.01 by the Wilcoxon rank-sum test. **(E)** Bar plots depicting relative abundances of bacterial taxa in the sham, SBI, BP, and combined groups. **(F)** Relative abundances of *Lactobacillus* among the sham, SBI, BP, and combined groups. **(G)** Relative abundances of *Allobaculum* among the sham, SBI, BP, and combined groups. **(H)** The differences of FITC-Dextran fluorescence intensity among the Sham, SBI, BP, and combined groups. **(I)** Representative images of occludin and claudin immunofluorescence staining in the colon and small intestinal tissues among the SBI, BP, and combined groups at 3 days. We demonstrated dramatically increased intestinal permeability **(H)** by a mechanism associated with reduced expression of epithelial tight junction proteins such as claudin and occludin **(I)**. This effect was completely restored by the oral administration of BP and probiotics. These data suggest that gut bacteria are involved in the control of intestinal permeability and in the occurrence of immune tolerance. *p < 0.05; **p < 0.01; and ***p < 0.001.

Compared with those in the SBI group, the IL-6, TNF-α, and IL-17 concentrations were markedly decreased postoperatively in the BP and combination groups at 1, 3, 7, and 14 days (Figure 3B; *P* < 0.05), thereby demonstrating that the oral administration of BP or BP with probiotics can decrease the concentrations of the proinflammatory cytokine IL-6, TNF, and IL-17.

Iba-1 and GFAP are important molecules of microglia and astrocytes, and their expression is closely related to the activation degree of the two types of glial cells. Compared with the SBI group, the intervention groups showed significantly reduced Iba-1 expression in activated microglia and thereby decreased nerve damage due to secondary inflammation. We determined the expression of GFAP in the surrounding peri-resection brain samples by immunofluorescence staining. We found that GFAP expression in the SBI group was significantly higher than those in the BP and combined groups (*P* < 0.05), similar to the Iba-1 results (Figure 3C), indicating that the oral administration of BP or BP combined with probiotics significantly reduced the activation of astrocytes and microglia. The comparison of Iba and GFAP between the BP and combined groups revealed that the expression levels of the two proteins were much lower in the combined group.

RETRACTED

The experimental results suggested that BP or BP combined with probiotics improved the conditions of the intestinal microbiota after SBI. The Chao1 indices in the SBI group were significantly lower than those in the sham, BP and combination groups at 3 days (*P* < 0 05; Figure 3D). After different oral interventions, we found that the genera of the microbiome were partially different between the BP and combined groups. In the BP group, *Lactobacillus* dominated, while in the combined group, in addition to *Lactobacillus*, *Allobaculum* increased markedly compared with the Sham, SBI groups (Figures 3E–G). We demonstrated dramatically increased intestinal permeability (Figure 3H) by detecting the FITC-dextran fluorescence intensity in the serum, which reflects the degree of damage to the intestinal barrier. At 3 and 7 days, the SBI group had the highest fluorescence concentration and the most serious intestinal damage. In the oral intervention group, the combined group showed the best recovery.

Moreover, the purely oral administration of probiotics achieved the desired effect in improving dysbiosis compared with that of the SBI group (Supplementary Figure 2).

Impaired immunological responses in the intestine are known to be associated with gut barrier dysfunction (Su et al., 2013). We investigated whether the oral administration of BP or probiotics combined with BP enhanced gut barrier function. Intestinal permeability was assessed by claudin and occludin expression in the colon and small intestine compared with that in the SBI group. Similarly, according to immunohistochemistry, the expression levels of the barrier-forming tight junction proteins claudin and occludin in the colon and small intestine were markedly higher. The protein expression levels of claudin and occludin were higher in the combined group than in the BP group (Figure 3I).

RETRACTED

### Immune Tolerance Induced by the Oral Administration of BP Through the IDO-AHR Pathway in the Gut

To investigate how the oral administration of BP or BP combined with probiotics induces immune tolerance, we performed quantitative proteomic analysis by TMT technology to explore the mechanism in the gut. In the BP vs. SBI group, there were 138 upregulated and 158 downregulated differentially expressed proteins (Figure 4A). The functions of these differentially expressed proteins were mainly binding, catalytic activity, structural molecule activity, transporter activity, and molecular function regulator. After Gene Ontology (GO) analyses of significantly differentially expressed genes, these differentially expressed proteins were shown to be mainly involved in cellular processes, metabolic processes, biological regulation, responses to stimuli, and regulation of biological processes (Figure 4B). *Via* KEGG pathway analysis, 10 metabolic pathways with statistical significance were identified (Figure 4C). Tryptophan metabolic pathways were selected to guide research on the mechanism. According to the tryptophan pathway, we wanted to determine how BPs and probiotics influence the intestine and brain.

**Figure 4:** IDO-AhR pathway in the gut of the BP group. **(A,B)** Volcano plot and heatmap of the differentially expressed proteins. **(C)** Associated signaling pathways. **(D–G)** The concentrations of metabolites of tryptophan. **(H)** The rate-limiting enzyme IDO1 in the colon and small intestine. **(I)** Representative images of AhR immunofluorescence staining in the colon and small intestinal tissues among the SBI, BP and combined groups at 3 days. *p < 0.05; ***p < 0.001; ns = not significant.

First, we tested metabolites, including 3-IPA, I-3CA, IAA, and kynurenine (Kyn), through metabolomics. The results showed that the concentrations of Kyn were strongly increased in the BP and combined groups at 3 days, while the concentrations of Kyn between the BP and combined groups were not significantly different (Figure 4D). The concentrations of 3-IPA and IAA demonstrated an opposite trend to I-3CA (Figures 4E–G). With respect to those of 3-IPA and IAA, the concentrations were apparently higher in the SBI group at 3 days, and the intervention measures had no obvious effects. In contrast, compared with those of the BP and combined groups, the concentration of I-3CA in the SBI group was decreased. In addition, there were no differences in Kyn, 3-IPA, I-3CA, or IAA between the PC and SBI groups (Supplementary Figure 3). Second, Trp metabolism through the Kyn pathway in the gut is mediated by the rate-limiting enzyme IDO1 and leads to the production of Kyn (Cervenka et al., 2017; Kennedy et al., 2017). We detected IDO, and the results suggested that the protein expression levels in the colon and small intestine were markedly lower in the SBI group at 3 days than in the BP and combined groups, according to western blot analyses, but the protein expression levels were not obviously different between the BP and combined groups (Figure 4H). Third, many indole derivatives, such as Kyn, indole-3-aldehyde (IAld), indole-3-acid-acetic acid (IAA), indole-3-propionic acid (IPA), indole-3-acetaldehyde (IAAld), and indole acrylic acid, are ligands for AhR (Hubbard et al., 2015b; Alexeev et al., 2018). Through immunohistochemistry, AhR protein expression was shown to vary. Compared to those in the BP and combined groups, the protein expression level was decreased in the SBI group; furthermore, AhR expression was higher in the combined group than in the BP group (Figure 4I).

RETRACTED

### Immune Tolerance Was Induced by the Oral Administration of Brain Protein Combined With Probiotics Through the IDO-AHR and TpH1–5-HT Pathways in the Brain

In the combined vs. BP group, a meaningful pathway was not found in the gut. Therefore, we performed quantitative proteomic analysis by TMT technology to explore the mechanism in the brain. In the combined vs. SBI group, there were 101 upregulated and 119 downregulated differentially expressed proteins (Figure 5A). The functions of these differentially expressed proteins included binding, catalytic activity, transporter activity, molecular function regulator, and structural molecule activity. GO analyses of significantly differentially expressed genes revealed that these differentially expressed proteins were mainly involved in cellular processes, biological regulation, regulation of biological processes, metabolic processes, and responses to stimuli (Figure 5B). *Via* KEGG pathway analysis, eight metabolic pathways that were significant were identified (Figure 5C). In the PC vs. SBI groups, the results showed that the serotonin pathway played a significant role in the mechanism (Supplementary Figure 4). Next, we tested the serum 5-HT concentration. Compared with those of the SBI and BP groups, the 5-HT concentration was markedly increased postoperatively in the combined groups at 1, 3, 7 and, 14 days (*P* < 0.05). Furthermore, the concentrations of 5-HT in the SBI and BP groups were significantly different on the 1st, 3rd, and 7th days (*P* < 0.05; Figure 5D). The concentration of 5-HT in the SBI group was higher than that in the BP group. The neurotransmitter 5-HT is produced in the brain through the Trp hydroxylase 2 enzyme (TpH2), where it plays an important role. This molecule is mostly produced in the gut and transported to the brain through peripheral blood. This process is catalyzed by the Trp hydroxylase 1 enzyme (TpH1). Thus, we detected TPH in the gut and brain through immunohistochemistry, and the TPH protein expression showed different levels. The expression of TPH was most obvious in the combined group, while in the SBI group, the expression of TPH was higher than that in the BP group (Figure 5E).

RETRACTED

**Figure 5:** The TpH1–5-HT pathway in the brain of the combined group. **(A,B)** Volcano plot and heatmap of the differentially expressed proteins. **(C)** Associated signaling pathways. **(D)** Comparison of 5-HT expression among the SBI, BP, and combined groups at 1, 3, 7, and 14 days. **(E)** The rate-limiting enzyme TPH in the colon, small intestine, and brain. *p < 0.05, **p < 0.01.

## Discussion

Cellular inflammatory reactions caused by brain trauma, neurosurgery, spontaneous cerebrospinal meningitis, and other sources of insult could worsen cerebral edema, thereby leading to irreversible neurological deficits. Studies have shown that the control of secondary immune damage can significantly reduce the volume of cerebral edema (Fu et al., 2015). Immune privilege in the gut is the result of a complex interplay among the gut microbiome, gut luminal antigens, and the intestinal epithelial barrier. Thus, the concept of the brain-gut-microbiota axis (BGMAx) provides a comprehensive picture of this relationship as follows: (1) neurotrauma results in local inflammation in the brain, which induces microglial priming (Kumar and Loane, 2012); (2) primed microglia increase the brain’s vulnerability to exaggerated immune responses to future external (e.g., subsequent TBI) or internal (e.g., infection) insults (Witcher et al., 2015); (3) TBI can cause structural and functional damage to the GI tract (Kharrazian, 2015); (4) this type of intestinal barrier dysfunction typically leads to increased intestinal permeability (Bischoff et al., 2014); (5) increased intestinal permeability is associated with a systemic immune response; and (6) the systemic inflammatory response emanating from the damaged gut can affect the vulnerable and previously primed microglia to further exacerbate neuroinflammation (Palin et al., 2008; Cunningham, 2013; Kelly et al., 2015).

First, we found that the gut microbiome was dramatically shifted in the patients with TBI and in the SBI group of rats at 3, 7, and, 14 days. The gut dysbiosis in TBI or SBI observed in our study was obvious and echoes the findings of previous reports. Nevertheless, in this study, the gut microbiome in TBI or SBI clearly deviated from that in the controls and showed very little overlap, indicating severe dysbiosis in brain injury. More interesting were the dysbiosis patterns, in which *Faecalibacterium* was depleted, whereas *Enterococcus*, *Parabacteroides*, and *Lachnoclostridium* were enriched in TBI. The microbiota profile of SBI was also altered, and *Lactobacillus* was enriched in the sham group. *Faecalibacterium, Lactobacillus*, and *Bifidobacterium* are involved in producing intestinal epithelial nutrition, maintaining immune homeostasis, and strengthening intestinal barrier functions. *Enterococcus* and *Parabacteroides* are mainly opportunistic pathogens and are associated with chronic inflammatory conditions and brain injury outcomes.

RETRACTED

We performed a series of experiments to observe the alteration of the barrier-forming tight junction proteins occludin and claudin in the intestine and the activation of Iba and GFAP in the brain after SBI at 3, 7, and 14 days through immunofluorescence and immunohistochemistry. The results identified dysbiosis as a key factor for damage to the intestinal mucosa and aggravated brain injury. One possible mechanism through which this occurs might be gut barrier destruction and the translocation of pathogenic bacteria from the gut to the blood, causing abnormal immune responses, which aggravate secondary immune damage to the brain. Our study proposed that a “brain-gut-microbiota” axis could play a crucial role in understanding SBI.

Second, we confirmed the establishment of immune tolerance through the oral administration of BP or BP combined with probiotics and evaluated their therapeutic effect. We repeatedly investigated the intestinal barrier and activation of astrocytes and microglia and assessed the alteration of dysbiosis after induction of immune tolerance among the SBI, BP, and combined groups. These results strongly demonstrated that the oral administration of BP or BP combined with probiotics can induce immune tolerance. However, the oral administration of a combination of BP and probiotics was better than the oral administration of pure BP in inducing immune tolerance and decreasing secondary inflammatory reactions. Houlden et al. (2016) showed that TBI affects the composition of the gut microbiota in the cecum and drew a link between TBI severity and changes in the microbiome, specifically in the composition of Bacteroidetes, Porphyromonadaceae, Firmicutes, and Proteobacteria. These conclusions coincide with our 16SrRNA results. In the TBI group, *Enterococcus* (Firmicutes phylum) predominated, and in the SBI group, *Bacteroides* predominated. Commensals influence gut-associated lymphatic tissue (GALT) formation, the induction of Peyer’s patches, and the induction of mucosal T cells and IgA plasma cells. The microbiota can induce proinflammatory and antiinflammatory responses. Germ-free mice have been shown to have decreased cellularity and functionality of the small intestine immune system with fewer plasma cells and intraepithelial lymphocytes, lower IgA levels, smaller Peyer’s patches, decreased lamina propria CD4+, and intraepithelial CD8αβ+ cells and increased susceptibility to pathogenic bacteria (Sommer and Bäckhed, 2013; Caricilli et al., 2014; Hörmann et al., 2014; Carabotti et al., 2015; Kubinak et al., 2015). Germ-free mice also lack Th17 cells, i.e., a subset of CD4+ T cells that secrete IL-17, which are a prominent T cell population found in the intestinal lamina propria that help maintain intestinal homeostasis by improving barrier function, stimulating mucin production, and affecting tight junction functionality and IgA transport (Caricilli et al., 2014). Disturbances of the BGMAx are implicated in many neurologic disease processes. Furthermore, the relatively recent discovery of the significance of the gut microbiota in BGMAx has led to a reevaluation of CNS diseases.

RETRACTED

Third, the mechanism of immune tolerance was proven (Figure 6). The results of the gut and brain proteomics suggested that the IDO-AhR pathway was affected by BPs, while the IDO-AhR and TpH1-5-HT pathways played important roles following treatment with BPs combined with probiotics. Endogenous tryptophan (Trp) metabolites have an important role in mammalian gut immune homeostasis. In the gut, Trp metabolism follows three major pathways in the gastrointestinal tract: (1) the direct transformation of Trp into several molecules, including ligands of the aryl hydrocarbon receptor (AhR), by the gut microbiota (Zelante et al., 2013); (2) the Kyn pathway (KP) in both immune and epithelial cells *via* indoleamine 2,3-dioxygenase (IDO) 1 (Clarke et al., 2013); and (3) the serotonin (5-hydroxytryptamine [5-HT]) production pathway in enterochromaffin cells *via* Trp hydroxylase 1 (TpH1; Yano et al., 2015). The comprehensive metabolic pathways of Trp provide key targets for us to reveal the mechanism of action.

**Figure 6:** Schematic representation of the mechanism involved in BP combined with probiotics inducing immune tolerance through the tryptophan pathway. Left part: the SBI model of rats showing dysbiosis, destruction of the intestinal barrier and tryptophan metabolism alterations. Right part: the interventions, the oral administration of BP combined with probiotics, triggered two different pathways in tryptophan metabolism. (1) The results of the BP intervention (red arrow) showed enrichment of *Lactobacillus*, which improved intestinal tight junctions and strengthened the IDO-AhR pathway. The pathway produced more Kyn, which was transported into the CNS to exert a protective influence on the brain. (2) The results of probiotic intervention (green arrow) demonstrated increased *Allobaculum*, which strengthened the TpH1–5-HT pathway. The neurotransmitter 5-HT alleviates depression after TBI and mitigates neurological impairment.

RETRACTED

The oral administration of BP can protect the mucosa and improve the condition of the intestinal microbiome while suppressing activated microglia and astrocytes. Metabolomic analysis has revealed that gut bacteria impact host immunity through a variety of metabolites, including indole metabolites (Wikoff et al., 2009), which originate from the microbial metabolism of tryptophan. AHR is a ligand dependent transcription factor activated by a variety of synthetic and biological molecules that plays an important role in immunological response and inhibition of inflammation (Hubbard et al., 2015a). The results of gut proteomics between the BP and SBI groups suggest that Trp metabolism-produced Kyn in the gut is catalyzed by the rate-limiting enzyme IDO1. The key role of the gut microbiota in stimulating IDO1 activity has been clearly demonstrated. Kyn, as a ligand of AhR, activates the IDO-AhR pathway, which plays an important role in the regulation of a number of host biological processes involving inflammatory suppression and immune tolerance. Specifically, Kyn, as a neurotransmitter, is transported to the central nervous system (CNS) *via* peripheral blood. Kyn is further metabolized into other metabolites, such as neuroprotective kynurenic acid and neurotoxic quinolinic acid, by kynurenine aminotransferase (KAT) and kynurenine 3-monooxygenase (KMO), respectively (Guillemin et al., 2005).

We continued to explore the pathways of the brain proteomics between the combined and SBI groups, and the serotonin metabolic pathway of brain proteomics was emphasized; thus, we believe that immune tolerance induced by BPs combined with probiotics is mediated *via* the serotonin metabolic pathway.

The gut microbiota is a major actor in intestinal 5-HT production (Yano et al., 2015). Its role has been demonstrated in germ-free mice that exhibit impaired 5-HT production in the colon and low 5-HT concentrations in the blood. According to the results of gut microbiota after the oral administration of BP or BP combined with probiotics, *Lactobacillus* and *Allobaculum* play important roles in the serotonin metabolic pathway.

As the blood-brain barrier breaks down after SBI, peripheral 5-HT enters the brain. Under normal conditions, the serotonin-selective reuptake transporter (SERT; encoded by the SLC6A4 gene) acts as a sponge to remove 5-HT from the interstitial space after production by ECs. This pivotal molecule involved in the local regulation of 5-HT availability is also responsible for 5-HT reuptake in the brain. Depression following TBI may exacerbate neuropsychological impairment and delay cognitive recovery (Hubbard et al., 2015a). Serotonergic antidepressants can treat depression following TBI (Fann et al., 2009; Jorge et al., 2016; Yue et al., 2017). Serotonin signaling plays an important role in the inflammatory response of secondary brain injury. It can inhibit the activation of astrocytes and microglia, thereby reducing the damage of inflammatory response (Ledo et al., 2016).

RETRACTED

In addition to its role as a neurotransmitter that regulates cognition, emotion, pain, and sleep, serotonin regulates cell division, differentiation, migration, myelination, synaptogenesis, and dendritic pruning during early brain development.

## Data Availability Statement

The raw data supporting the conclusions of this article will be made available by the authors, without undue reservation.

## Ethics Statement

The animal study was reviewed and approved by IACUC committee of Tianjin Key Laboratory of Cerebral Vascular and Neurodegenerative Diseases, China.

## Author Contributions

HY, LX, and XT designed the study. YH, SS, QW, and WF accomplished the SBI model, specimen acquisition, and inmunefluoresence staining. YH and SS performed data analysis. YH and LX wrote the manuscript. All authors contributed to the article and approved the submitted version.

## Conflict of Interest

The authors declare that the research was conducted in the absence of any commercial or financial relationships that could be construed as a potential conflict of interest.

## Abbreviations

Iba: Ionized calcium binding adaptor molecule
GFAP: Glial fibrillary acid protein
IDO: Indoleamine 2,3 dioxygenase
AhR: Aryl hydrocarbon receptor
TpH1: Tryptophan hydroxylase 1
BGMAx: Brain-gut-microbiota axis
5-HT: 5-hydroxytryptamine
TBI: Traumatic brain injury
SBI: Surgical brain injury
Trp: Tryptophan
Kyn: Kynurenine
TMT: Tandem mass tag
3-IPA: Indole-3-propionic acid
I-3CA: Indole-3-carboxaldehyde
IAA: Indole-3-acid-acetic.
